# Analysis and Research on Audience Satisfaction of Performing Arts Projects in Tourist Scenic Spots Based on the ASCI Model and Big Data

**DOI:** 10.1155/2022/5907900

**Published:** 2022-05-23

**Authors:** Jiaran Ding, Lin Yu

**Affiliations:** ^1^Chengdu Jincheng College, Chengdu 611731, China; ^2^Jiangxi University of Technology, Nanchang 330098, China; ^3^SEGi University, Kuala Lumpur 47810, Malaysia

## Abstract

The development trend of tourism performance networking, although convenient for audience consumption, also makes the performance information present the development trend of big data. In the mass of information, how to accurately locate products and improve audience satisfaction is an urgent problem to be solved. In order to better explore the evaluation of tourism performance by the customer satisfaction evaluation model, analyze the development prospect of tourism in Jiangxi Province in the future, improve the customer satisfaction evaluation model with rough set, and propose a composite customer satisfaction evaluation model. By setting the adjustment value of the evaluation index, the model not only avoids the “false eigenvalue” of the satisfaction evaluation result but also simplifies the calculation process of the model and improves the accuracy, calculation efficiency, and single data processing capacity of the satisfaction evaluation. According to the MATLAB simulation results, the composite customer satisfaction evaluation model constructed in this study is better, the calculation accuracy is >97%, and the calculation time is 40 seconds, which are better than the original customer satisfaction evaluation model. Therefore, the composite customer satisfaction evaluation model can be applied to the evaluation of tourism performance products to provide data support for the evaluation price of audience satisfaction in Jiangxi Province.

## 1. Introduction

Tourism performance is not only an important part of social entertainment [1] but also an important part of local GDP. However, tourism performance information presents the development trend of big data, and the original genetic, Bayesian, and other algorithms cannot accurately evaluate satisfaction. There is an urgent need for an adaptive improved algorithm to solve the problem of massive data processing and optimize the evaluation process of satisfaction [2]. In addition, the emergence of information technologies such as big data, Internet of things, and cloud platform increases the complexity of audience analysis and the difficulty of satisfaction evaluation [3]. The original customer satisfaction evaluation model mainly analyzes a small amount of data and lacks the analysis of massive data and multiattribute data [4]. Therefore, it is the focus of attention and research to improve the customer satisfaction evaluation model and put forward a model that meets the needs of tourism performance analysis. Based on the above background, this study proposes a composite customer satisfaction evaluation model to analyze the tourism performance in Jiangxi Province and judge the satisfaction of the audience. At present, in the process of audience satisfaction analysis, there are some problems, such as large amount of data, unsatisfactory processing effect of the original model, and inaccurate analysis results. Audience satisfaction analysis needs a suitable algorithm as an aid, in order to better analyze. The ASCI model can make quantitative and qualitative analyses of audience satisfaction and combine with relevant data to make comprehensive analysis. Compared with other methods, the calculation process of the ASCI model is simpler and the calculation effect is better. ASCI is suitable for the field with less data and complex data structure, while the data processing of audience satisfaction survey is difficult, so it is suitable for the ASCI model. The ASCI model itself also has some deficiencies, which need to be further improved. It should be combined with cluster analysis and constraint function to make up for the shortcomings of its own construction and improve the application effect of the model. According to the development background of big data, this study proposes a comprehensive customer satisfaction evaluation model to analyze the performance of tourism in Jiangxi Province and judge the satisfaction of visitors.

## 2. Literature Review

The American customer satisfaction index model is a comprehensive model first proposed by Fornell et al. The model has been improved and improved by Sweden, Europe, and other countries. It has become a global classic model and is widely used in various fields of society [5]. The American customer satisfaction index model takes customer expectation as the starting point and customer satisfaction as the focus to analyze customer perception, perceived value, perceived complaint, and customer loyalty [6]. The American customer satisfaction index model was first applied to hotel management and was introduced to China in 1999. The American customer satisfaction index model belongs to the category of the comprehensive analysis algorithm. It uses questionnaires, interviews, and other forms to obtain data and makes qualitative and quantitative analyses [7].Tourism performance projects are networked, digital, and multidimensional. The original American customer satisfaction index model cannot meet the requirements and deal with a large amount of passenger information [8]. There are problems such as inaccurate results, prolonged processing time, and many processing times. The rough set is a fuzzy analysis method, which realizes the estimation and budget of data, finds out the characteristic data from the massive data, and achieves the purpose of reducing the data scale [9]. At present, the rough set is widely used in the field of big data analysis, which can filter big data and improve the calculation accuracy [10]. In addition, increasing the threshold in the rough set can adjust the calculation accuracy and meet the needs of different calculation models. Therefore, based on the American customer satisfaction index model, this study takes customer expectation, satisfaction, customer complaint, loyalty, and perceived value as indicators and combines rough set theory to analyze the tourism performance in Jiangxi Province. The validity of the model is verified by simulation analysis, and the processing ability of the model to massive audience data is judged.

## 3. Methods

### 3.1. Description of the American Customer Satisfaction Index Model

ASCI is a comprehensive analysis model, which can make qualitative investigation and quantitative analysis on audience satisfaction. It was first used in the art field and then gradually adopted by computer, engineering, and network fields. This method judges and analyzes satisfaction by collecting multiangle data. The description of the American customer satisfaction index model takes customer satisfaction as the ultimate goal and customer expectation as the starting point. The indicators of perceived quality, perceived value, customer complaint, and customer loyalty in the model are variable indicators [11], which will be affected by market, industry, policy, and other factors. The American customer satisfaction index model enriches the European customer satisfaction index model and perfects the Swedish customer satisfaction index model, which is a comprehensive model [12]. Among the indicators, customer perception, customer quality, and customer loyalty are the key indicators, and customer complaints are auxiliary indicators. The American customer satisfaction index model simplifies the complex indicators [13], combines the contents of similar indicators, defines the role of customers, and realizes dynamic analysis. Compared with other models, the index of the American customer satisfaction index model is more comprehensive, the evaluation process is simpler [14], and the analysis dimension is reduced, which is suitable for diversified customer satisfaction analysis. However, the American customer satisfaction index model is easy to fall into local extremum, and about 2–8% of the results are local extremum, which affects the accuracy of satisfaction evaluation. In addition, the American customer satisfaction index model only analyzes the original data [15] and cannot estimate and judge the data, which further reduces the accuracy of the results. As the customer complaint index is a dynamic index, it has an obvious impact on customer satisfaction, so it needs to be calculated for many times to prolong the calculation time. At the same time, the initial index of the American customer satisfaction index model is customer expectation. Under the big data, the calculation complexity of this index will increase by 20–30%, further prolonging the calculation time. In this study, rough set theory is introduced to preprocess customer expectations, and qualitative analysis is carried out on indicators such as perceived value, perceived quality, customer complaint, and customer loyalty, so as to improve the shortcomings of the original model. The specific model principle is shown in Figure 1.

As can be seen from Figure 1, there are many data design contents in ASCI, including not only the prediction value, user understanding, and prediction quality but also constructing satisfaction set and understanding set and incorporating big data information.

### 3.2. Determine the Indicators of the Customer Satisfaction Index Model

The selection of indicators should be from four aspects: perceived quality, perceived value, customer complaint, and customer loyalty. The content of indicators should be evaluative and predictive. Reasonable indicators can simplify the analysis process and realize multidimensional calculation. Because the customer satisfaction index model needs to deal with network big data, it should not only realize the calculation of a single index but also calculate the relationship between different indexes, so the selection of indexes should be more rigorous. Tourism performance products belong to a dynamic process, which are affected by local policies, economy, geographical location, and other factors, as well as their own reputation, reputation, brand, and service. In order to better model risk, each index should integrate 4-5 factors and integrate threshold and weight to form a multiangle analysis. In addition, the setting of threshold and weight can reduce the occurrence rate of local extremum and realize the global analysis of each index. According to the above analysis, this study puts forward the input index hypothesis. Hypothesis 1: the input index of the customer satisfaction index model is *x*_i_ and the output index is *y*_i_. The input indicators of different dimensions are *x*_*ij*_ and the output indicators are *y*_*ij*_, where *i* and *j* belong to the set (1, 2,…, *n*). Then, the relationship between the input index *x*_*ij*_ and the output index *y*_*ij*_ is

(1) $$\begin{array}{c} y_{ij}=\sum_{i,j=1}^{n}\frac{\left(x_{ij}-x_{i-1j-1}\right)}{{\bar{y}}_{ij}+\mu }, \end{array}$$

where *μ* is the adjustment index of the customer satisfaction index model, ${\bar{y}}_{ij}$ is the average value of output indicators and the average value of industry satisfaction, (*x*_*ij*_ − *x*_*i*−1*j*−1_) is the difference of different input indicators, representing the improvement degree of evaluation indicators, and ∑_*i*,*j*=1_^*n*^(*x*_*ij*_ − *x*_*i*−1,*j*−1_) is the sum of all input indicators and represents the overall value of the input indicators.

### 3.3. The Rough Set Theory

Because the audience data of the customer satisfaction index model is large and affected by many factors, the calculation process is complex.

In order to realize the processing of massive audience data, rough set analysis should be carried out to eliminate irrelevant data and improve the single data processing capacity as much as possible. Hypothesis 2: the Euclidean distance between any audience data is q, and the shortest distance between the two data is taken as the input value. In this case, the rough set only needs to judge the distance between any data, include the qualified data, and eliminate other data. In order to facilitate later calculation, the included data are defined as 1 and the excluded data are defined as 0 In order to ensure the accuracy of calculation and avoid the problem of local extreme value, the calculation direction of data shall be specified. Hypothesis 3: if the distance between any data is the smallest and the calculation direction is positive, the data will be included; otherwise, the data will be eliminated. According to assumptions 2 and 3, the calculation formula of the distance between any data can be obtained, as shown in the following equation.

(2) $$\begin{array}{c} S_{ij}=\left\{\begin{array}{c} \frac{\sqrt{p{\left(x_{ij},y_{ij}\right)}^{2}+q{\left(x_{ij},y_{ij}\right)}^{2}}}{\left\{\bar{q\left(x_{i},y_{i}\right)},\bar{p\left(x_{j},y_{j}\right)}\right\}}\\ \Delta \overset{⟶}{p\left(x_{ij},y_{ij}\right)}+\Delta \overset{⟶}{q\left(x_{ij},y_{ij}\right)}+\frac{1}{\xi } \end{array}\right., \end{array}$$

where *p*(*x*_*ij*_, *y*_*ij*_) is the abscissa between any two data under big data, *q*(*x*_*ij*_, *y*_*ij*_) is the ordinate between any two data, $\left\{\bar{q\left(x_{i},y_{i}\right)},\bar{p\left(x_{j},y_{j}\right)}\right\}$ is the average value set between any two data, $\Delta \overset{⟶}{p\left(x_{ij},y_{ij}\right)}$ is the abscissa direction of any two data, $\Delta \overset{⟶}{q\left(x_{ij},y_{ij}\right)}$ is the ordinate direction of any two data, and 1/*ξ* is the adjustment function of the direction. Because each customer has different expectations and complaints, it is necessary to set dynamically, that is, increase the threshold and weight. Hypothesis 4: if the dynamics between any two data is Q and is affected by the threshold m and weight *w*, the calculation of dynamics is

(3) $$\begin{array}{c} Q_{ij}=\sqrt{\sum_{i,j=1}^{n}\underset{x⟶\infty }{\lim}\omega_{ij}\cdot {\left[m_{ij}-\frac{1}{\underset{x⟶\infty }{\lim}\left(m_{ij}\right)}\right]}^{2}}\cdot \tau , \end{array}$$

where *ω*_*ij*_ is the weight of any data under big data, *m*_*ij*_ is the threshold of any data under big data, *τ* is the adjustment coefficient of weight and threshold to ensure that the weight and threshold are between 0 and 1, and $\left[m_{ij}-1/\underset{x⟶\infty }{\lim}\left(m_{ij}\right)\right]$ is the variation difference of the threshold to ensure the direction of the threshold. After calculating the dynamics of the data *Q*_*ij*_, assign a value to it. According to rough set theory, *m* = 1 and *w* = 0 can be made, and progressive analysis can be carried out gradually.

### 3.4. Construction of the Composite Customer Satisfaction Index Model

The analysis of customer satisfaction is a gradual process. It is necessary to eliminate the audience data in multiple dimensions and select the data values that meet the requirements. The whole calculation process is the traversal process of all data, and multidimensional data traversal is required. In order to reduce the number of traversals, the audience data should be predicted. In this process, it is necessary to avoid falling into local extremum and ensure that the calculated data is global extremum. Meanwhile, in the process of model analysis, the influence of big data on the results should be reduced to ensure the stability of the calculation results. On the basis of referring to relevant domestic models, this study integrates weight, threshold, and rough set theory. Hypothesis 4: under big data, if the satisfaction output is *y*_*ij*_, the actual calculation result is *o*_*ij*_, the estimated result is *r*_*ij*_, and the calculation of the result is

(4) $$\begin{array}{c} y_{ij}=\left\{\begin{array}{c} o_{ij}=\sum_{i,j=1}^{n}\left[w_{ij}\cdot m_{ij}\cdot f\left(x_{ij}+y_{ij}\right)\right]\\ r_{ij}=\left[\sum_{i,j=1}^{n}w_{ij}\cdot m_{ij}\cdot F\left(\Delta x_{ij}+\Delta y_{ij}\right)\right]+\psi \end{array}\right., \end{array}$$

where *f*(*x*_*ij*_+*y*_*ij*_) is the actual calculation result, *F*(Δ*x*_*ij*_+Δ*y*_*ij*_) is the result of estimation by difference, and *ψ* is the adjustment coefficient in the estimation to ensure that the estimation is within a reasonable range. Similarly, the adjustment coefficient is also affected by policies, marketing means, data volume, industry environment, and other factors, which belongs to dynamic variation. Then, the adjustment coefficient *ψ* is calculated as

(5) $$\begin{array}{c} \psi =\frac{1}{\eta }\sum_{i,t=1}^{n}\left\{\left[g\left(x_{ij}\right)-S_{i}]-]z\left(y_{ij}\right)-S_{j}\right]\right\}, \end{array}$$

where *g*(*x*_*ij*_) is the adjustment function of the input index *x*_*ij*_, *z*(*y*_*ij*_) is the adjustment function of *y*_*ij*_, *S*_*i*_ is the average level of each index *i*, *S*_*j*_ is the average level of different factors *j*, and *η* is the local adjustment coefficient. The adjustment coefficient *ψ* belongs to the macro adjustment coefficient, which is inversely proportional to the local adjustment coefficient*η*. In order to ensure the accuracy of the adjustment coefficient *g*(*x*_*ij*_) and *z*(*y*_*ij*_), it is necessary to transpose and express them with *g*(*x*_*ij*_)^*T*^ and *z*(*y*_*ij*_)^*T*^. Because the customer satisfaction index model belongs to a gradual analysis process, it should be calculated iteratively and finally get the expected results. Hypothesis 6: if the horizontal iteration result is *E*_*i*_ and the vertical iteration result is *E*_*j*_, the calculation process of the input index is

(6) $$\begin{array}{c} \left\{\begin{array}{c} E_{i}=\frac{\left[\sum_{i,j=1}^{n}\Delta x_{ij}\right]}{\bar{\underset{x⟶\infty }{\lim}f\left(x\right)}}w_{ij}m_{ij}\\ E_{j}=\frac{\left[\sum_{i,j=1}^{n}\Delta y_{ij}\right]}{\bar{\underset{y⟶\infty }{\lim}F\left(y\right)}}w_{ij}m_{ij} \end{array}\right., \end{array}$$

where $\underset{x⟶\infty }{\lim}f\left(x\right)$ is the maximum horizontal coordinate of any data, $\underset{y⟶\infty }{\lim}F\left(y\right)$ is the maximum ordinate of any data, Δ*x*_*ij*_ is each progressive quantity of abscissa, and Δ*y*_*ij*_ is each increment of the ordinate. The whole gradual process is shown in Figure 2.

It can be seen from Figure 2 that the passenger data gradually approaches the actual (*E*_*i*_, *E*_*j*_), and this process is a gradual process, which needs continuous optimization and analysis.

### 3.5. Calculation Steps of the Composite Customer Satisfaction Index Model

The integration of the rough set and customer satisfaction index model not only reduces the occurrence rate of local extremum but also improves the depth of audience data mining and more comprehensively analyzes tourism performance products [16]. In addition, in the process of multiple iterations, the change range of the analysis results is smaller, and the gap between the analysis results and the reality is smaller. The composite customer satisfaction index model is divided into the steps shown in Figure 3.

## 4. Results and Discussion

This study takes the tourism performance project in Jiangxi Province as the research object, analyzes the satisfaction of its online audience, and verifies the effectiveness of the composite customer satisfaction index model.

### 4.1. The Sample Object

Make a comprehensive analysis based on the audience data from 2019 to 2020. The data come from Jiangxi Provincial Tourism Administration. The data include Jinggangshan in Ji'an, dream home in Wuyuan, Longhu Mountain in Yingtan, Peony Pavilion in Fuzhou, Sanqingshan Mountain, eternal love of the bright moon in Yichun, and Ruijin in blood bath in Ganzhou. The statistical indicators are as follows: x1 perceived quality (unit: none), x2 perceived value (unit: none), x3 customer complaint (unit: %), and x4 customer loyalty (unit: %), as given in Table 1.

It can be seen from Table 1 that the aggregation degree of different input indicators and transfer factors is greater than 95% and higher than the global threshold of 0.98. The data of sports economic industry meet the specific requirements and can be analyzed and calculated. According to the survey of tourism performance projects in Jiangxi Province given in Table 1, it can be seen that the satisfaction iterative centers (Ei, Ej) mainly focus on (0.55, 0.39). Moreover, there are three forms of data acquisition, including questionnaire (reliability and validity >7.2, and the recovery rate is 98%), actual interview, and big data. The proportion of various data is given in Table 2.

### 4.2. Accuracy of the Composite Customer Satisfaction Index Model

Compared with the customer satisfaction index model, the accuracy of the composite customer satisfaction index model is higher, which can reach more than 97%, as shown in Figure 4.

As can be seen from Figure 4, the accuracy of the composite customer satisfaction index model is between 98% and 99%, while the accuracy of the original customer satisfaction index model is between 92% and 96%, and the change range of accuracy and results are better than that of the original customer satisfaction index model. The reason for the above problems is that the composite customer satisfaction index model uses the rough set for big data preprocessing to eliminate irrelevant audience data and reduce the impact of irrelevant data on the results and the amount of performance data. In addition, the fusion of threshold and weight greatly reduces the occurrence rate of local extremum. At the same time, the calculation results proposed in this study still have a certain range, mainly due to the prediction results in the calculation process [17].

### 4.3. Local Extremum of the Composite Customer Satisfaction Index Model

The calculation direction is the criterion for judging the extreme value. The calculation direction of the composite customer satisfaction index model is shown in Figure 5.

It can be seen from Figure 5 that there is a certain angle between the calculation direction and positive direction of the composite customer satisfaction index model, mainly due to the deviation in the setting of threshold and weight during the calculation process. However, the overall calculation direction of the composite customer satisfaction index model is the same, which shows that the model has a good control effect on the calculation direction and greatly reduces the occurrence rate of local extreme values, and meets the requirements of audience satisfaction evaluation under the condition of big data。

### 4.4. Calculation Time of the Composite Customer Satisfaction Index Model

Calculation time is not only an important index to improve audience satisfaction but also the basis of model analysis. Under the same amount of data, compare the calculation time of different models, and the results are shown in Figure 6.

As can be seen from Figure 6, the calculation time of the composite customer satisfaction index model is better, which is significantly lower than that of the original customer satisfaction index model. The calculation time of the former is less than 40 seconds and that of the latter is less than 55 seconds. In the process of 0–5 iterations, the calculation time of the two models is similar, which shows that the calculation time of the two models is the same under the amount of data, and also verifies the effectiveness of the original customer satisfaction index model. However, in 5–25 iterations, the calculation time of the composite customer satisfaction index model is significantly reduced. Due to the original customer satisfaction index model [18], it shows that the composite customer satisfaction index model is suitable for big data analysis. Therefore, the composite customer satisfaction index model can realize the analysis of audience satisfaction under big data in the analysis of tourism performance products in Jiangxi Province.

## 5. Conclusion

The composite customer satisfaction index model realizes the analysis of audience big data through rough set theory, simplifies the calculation process, increases the amount of single processing data, and shortens the calculation time by means of prediction and judgment. Under big data, by setting the threshold and weight, the occurrence rate of local extreme value is reduced and the accuracy of calculation is improved. The ASCI model can better evaluate audience satisfaction and lay a foundation for improving audience satisfaction. The ASCI model has better comprehensive analysis results and higher analysis ability. The simulation results show that the calculation accuracy of the composite customer satisfaction index model is more than 98% and the calculation time is less than 40 seconds, which is significantly better than the original customer satisfaction index model. Therefore, the model proposed in this study is better under big data, which can provide support for the evaluation of audience satisfaction in Jiangxi Province and promote the development of local tourism performance. In addition, there are still some deficiencies in the research process of this study, mainly reflected in the data structure, and the structured data and semistructured data in big data are not analyzed under big data. Generally speaking, semistructured data in big data account for a large proportion and have a great impact on customer satisfaction. There are still some shortcomings in the research of this study; in the future research, the data structure will be analyzed to further improve the accuracy of audience satisfaction evaluation.

## Figures and Tables

**Figure 1:** The American customer satisfaction index model under the background of big data.

**Figure 2:** The gradual process of the customer satisfaction index model under big data.

**Figure 3:** The calculation process of the composite customer satisfaction index model.

**Figure 4:** The evaluation accuracy of audience satisfaction under different models.

**Figure 5:** The calculation direction of audience satisfaction.

**Figure 6:** The calculation time of different methods.

**Table 1:** The survey data of tourism performance projects in Jiangxi Province.

The place	The content	The number of evaluation indicators (piece)				*E*_*i*_	*E*_*j*_
		x1	x2	x3	x4		
Ji'an	“Jinggangshan”	14	7	6	21	0.57	0.33
Wuyuan	“Home in a dream”	12	8	22	8	0.51	0.33
Yingtan	“Longhu Mountain in search of dreams”	14	5	11	23	0.23	0.42
Fuzhou	“Dream seeking Peony Pavilion”	19	19	21	14	0.49	0.48
Mount Sanqingshan	“The world is clear”	12	19	9	22	0.42	0.42
Yichun	“Eternal love of the bright moon”	20	11	16	11	0.46	0.37
Ganzhou	Ruijin in blood bath	17	13	17	9	0.51	0.35

**Table 2:** The proportion of different audience data.

The place	The content	The questionnaire	The interview	The big data
Ji'an	“Jinggangshan”	20.2	50.4	29.4
Wuyuan	“Home in a dream”	20.2	40.323	39.5
Yingtan	“Longhu Mountain in search of dreams”	50.4	30.2	19.4
Fuzhou	“Dream seeking Peony Pavilion”	30.2	20.2	49.6
Mount Sanqingshan	“The world is clear”	20.2	70.6	9.3
Yichun	“Eternal love of the bright moon”	20.2	40.3	39.5
Ganzhou	Ruijin in blood bath	30.2	60.5	9.3

## Data Availability

The data used to support the findings of this study are available from the corresponding author upon request.
